The article "Bionic Nonsmooth Drag Reduction Mathematical Model Construction and Subsoiling Verification" was published in 2021. Journal: Appl Bionics Biomech.

# Bionic Nonsmooth Drag Reduction Mathematical Model Construction and Subsoiling Verification

**DOI:** 10.1155/2021/5113453

**Published:** 2021-11-20

**Authors:** Baoguang Wu, Ruize Zhang, Pengfei Hou, Jin Tong, Deyi Zhou, Haiye Yu, Qiang Zhang, Jinsong Zhang, Yuelin Xin

**Affiliations:** ^1^The College of Biological and Agricultural Engineering, Jilin University, 5988 Renmin Street, Changchun 130025, China; ^2^The Key Laboratory of Bionic Engineering, Jilin University, 5988 Renmin Street, Changchun 130025, China

## Abstract

In this study, a bionic nonsmooth drag-reducing surface design method was proposed; a mathematical model was developed to obtain the relationship between the altitude of the nonsmooth drag-reducing surface bulges and the spacing of two bulges, as well as the speed of movement, based on which two subsoiler shovel tips were designed and verified on field experiments. The mechanism of nonsmooth surface drag reduction in soil was analyzed, inspired by the efficient digging patterns of antlions. The nonsmooth surface morphology of the antlion was acquired by scanning electron microscopy, and a movement model of the nonsmooth surface in soil was developed, deriving that the altitude of the nonsmooth drag-reducing surface bulge is proportional to the square of the distance between two bulges and inversely proportional to the square of the movement speed. A flat subsoiler shovel tip and a curved tip were designed by applying this model, and the smooth subsoiler shovel tips and the pangolin scale bionic tips were used as controls, respectively. The effect of the model-designed subsoilers on drag reduction was verified by subsoiling experiments in the field. The results showed that the resistance of the model-designed curved subsoiler was the lowest, the resistance of the pangolin scale bionic subsoiler was moderate, and the resistance of the smooth surface subsoiler was the highest; the resistance of the curved subsoiler was less than the flat subsoilers; the resistance reduction rate of the model-designed curved subsoiler was 24.6% to 33.7% at different depths. The nonsmooth drag reduction model established in this study can be applied not only to the design of subsoilers but also to the design of nonsmooth drag reduction surfaces of other soil contacting parts.

## 1. Introduction

Soil structural degradation is believed to be one of the most severe forms of soil degradation from traditional farming practices, which refers to the reduction in porosity between soil clumps, commonly known as soil compaction [1]. When soil porosity is less than 0.2 to 0.3 mm, crop roots will have difficulty traveling freely through the soil, seriously affecting the uptake of soil nutrients and water by crop roots and reducing crop yields [2]. Soil structure degradation is a worldwide problem that causes enormous economic damage every year [3–5]. Due to soil structure degradation, losses reach $144 million in just one farming region of Australia annually; crop yield losses in the USA amounts to $1 billion a year [6].

The article "Bionic Nonsmooth Drag Reduction Mathematical Model Construction and Subsoiling Verification" was published in 2021. Journal: Appl Bionics Biomech.

Soil compaction is preventable and can be prevented at an early stage through less tillage, no tillage, and reducing the number of tractor entries [7]. Less or no tillage can preserve soil texture by promoting the development of soil biological populations while reducing soil disturbance [8, 9]. Even with minimum or no tillage, the increased number of tractor entries and the natural settlement of the more viscous soil particles can easily cause soil compaction, which can be severe enough to form a plow pan 20 to 30 cm below ground level. The plow pan generally presents a laminar structure, which is heavier than the typical tilled soil; its thickness is typically around 10 cm, with greater solidity, less porosity, poorer water permeability, and air permeability [10, 11].

At present, subsoiling is the fastest and most widespread method to break the plow pan and improve soil compaction. By loosening the soil without turning it over, subsoiling not only loosens the hard plow pan, regulates the ratio of soil solids, liquids, and air, creates a virtual and solid tillage structure, reduces soil erosion but also improves the fertility and moisture of the tillage layer. As a result, subsoiling technology can significantly increase crop yields in areas of soil compaction, especially for deep-rooted crops [12–15].

Unlike the traditional tillage method, the subsoiling depth is generally larger, with deeper soil penetration [16, 17]. Soil adhesion and subsoiling resistance are bigger; subsoiler shovel tip part is very easy to form a large piece of soil nucleus [18, 19], which not only leads to increased subsoiling energy consumption and poor subsoiling quality, and seriously subsoiling resistance increases sharply, directly affecting the routine operation or lead to the destruction of machinery [20]. This problem can be solved by vibration, electroosmotic and bionic methods [21–23]. Although vibration and electroosmotic methods can reduce soil adhesion and achieve the purpose of reducing resistance, they require additional mechanisms to achieve this, which not only makes the structure more complex but also causes additional energy consumption [24–26].

In recent years, the development of bionics has injected new vitality into agricultural machinery drag reduction technology [27–29]. Natural organisms have evolved excellent functions and unique geometric structures over billions of years, and among them, animals that are good at digging have evolved superior digging organs. These superior characteristics have been applied to the field of resistance reduction in agricultural machinery, and fruitful research results have been achieved [30, 31]. Li et al. [32, 33] studied the structural characteristics of the dung beetle's touching soil body surface and designed a convex bun type bionic plow, acquiring the efficiency of drag reduction 6.6% to 12.7% through soil bin tests. Ren [34] developed convex bun type and stripe type bionic pushing plates based on the structural characteristics of the dung beetle's head clypeus, which reduced resistance by 15% to 41%. Tong et al. [35] chose the mus musculus as the bionic prototype and obtained the paw contour equation through mathematical regression methods, thus establishing a mathematical model; Guo [36] applied the paw of the oryctolagus cuniculus to the design of subsoiler, and the bionic subsoiler could reduce resistance by 8.23% on average compared with traditional subsoilers. Despite the outstanding achievements of these bionic technologies, there is less research on the bionic drag reduction mechanism of agricultural machinery soil touching parts, especially in the field of bionic nonsmooth surface drag reduction; how to determine the quantitative relationship of nonsmooth surfaces key parameters is a problem which needs to be solved in this field.

The article "Bionic Nonsmooth Drag Reduction Mathematical Model Construction and Subsoiling Verification" was published in 2021. Journal: Appl Bionics Biomech.

In this study, the larvae of antlions, which are good at digging, were used as a bionic prototype. The antlions belong to the family of ant lacewings in the order Plecoptera. They show a spindle streamline shape, and their whole bodies are covered with nonsmooth structures. The antlion larvae are excellent at using the vibration of their hindquarters to make holes in the sand and create funnel traps to trap their prey [37]. The antlions' microstructure of the body surface was observed by scanning electron microscopy (SEM) and stereomicroscope; the external profile features were extracted, the traction force changes during the contact between the nonsmooth surface, and the soil was analyzed. Further, the quantitative relationship between the altitude of the bulge, the distance of two bulges, and the movement speed was established. This mathematical model was applied to design two types of subsoilers, planar, and curved, and the pangolin scale bionic subsoilers and smooth subsoilers were used as controls. It has been shown that pangolins are very good at digging, and the scales on their bodies help to improve their digging ability [38, 39]. Through field tests, the resistance of six types of subsoilers was compared, and the resistance reduction effect of nonsmooth surface subsoilers was tested, which verifies the mathematical model's correctness of nonsmooth resistance reduction surface. This is important for reducing the subsoiling resistance and improving the quality of subsoiling, as well as providing a model basis for the design of nonsmooth drag-reducing surfaces for the soil touching parts of agricultural machinery.

The article "Bionic Nonsmooth Drag Reduction Mathematical Model Construction and Subsoiling Verification" was published in 2021. Journal: Appl Bionics Biomech.

## 2. Construction of a Nonsmooth Drag Reduction Model for Soil Touching Parts

In this section, the nonsmooth body surface structure of antlions was obtained; a nonsmooth drag reduction mathematical model was constructed, which was applied to the design of the subsoiler shovel tips.

### 2.1. Acquisition of Antlions' Body Surface Structures

Three antlions were collected as specimens with an average length of 9.07 mm and a width of 3.86 mm (Guangdong, China). The overall structures of the antlions were obtained by a stereomicroscope (OLYMPUS SZX7, Olympus Optical Co., Ltd., Tokyo, Japan), and the surface microstructure was obtained with the SEM (Zeiss, EVO18, Carl Zeiss AG, Germany). The body surface structures are shown in Figure 1.

Antlions were covered with nonsmooth structures all over their bodies (Figure 1(a)). Based on statistics of the space between the camera and the surface of antlions' back, and the lengths of the antlions' back setae in the raised and depressed areas, it was determined that the spacing range of the antlions' back raised was 300 *μ*m to 500 *μ*m, with a variation in altitude ranging from 100 *μ*m to 200 *μ*m (Figures 1(g), 1(i), and 1(j)). Antlions were covered with setae all over their bodies, among which marginal setae aggregated and varied in length from 200 *μ*m to 700 *μ*m with a mean value around 500 *μ*m (Figures 1(d), 1(e), and 1(j)). The antlions' back raised construction and setae formed their submillimeter structure. In addition to the margins, the back, head, and tail of the antlions were also riddled with setae (Figures 1(f)–1(h)), which varied in altitude from 50 to 150 *μ*m, in spacing from 50 to 100 *μ*m, and had corrugated jaws (Figures 1(b) and 1(c)); these features constituted the nonsmooth surface structure at the micron scale. Further magnification of the body surface revealed a grooved structure (Figures 1(d) and 1(e)), with the width of the grooves varying in the range of 2-10 *μ*m and the altitude ranging from 0.5 *μ*m to 2 *μ*m. These features constituted a submicron nonsmooth structure. Together, the three scales of structure constitute the nonsmooth pattern of antlions. This feature assisted in causing significant soil disturbance while antlions were digging, reducing the resistance.

The article "Bionic Nonsmooth Drag Reduction Mathematical Model Construction and Subsoiling Verification" was published in 2021. Journal: Appl Bionics Biomech.

### 2.2. Construction of a Nonsmooth Drag Reduction Mathematical Model

The shear resistance of the soil is the main factor in the amount of resistance when the antlion makes holes in the soil. Since viscous material and water are present in the soil, the soil possesses a certain amount of shear resistance even without positive pressure. This force is known as cohesion, and cohesion and internal friction force together determine shear strength.  Figure 2 shows the correspondence between the positive pressure *F*, soil shear force *F*_*s*_, the cohesion *cA*, and the angle of internal friction *φ* [40].

In the environment where the antlions live, soil cohesion is low, and the shear strength of the soil is mainly determined by internal friction index *f*, which is strongly influenced by the loose index *K*_*S*_ of the soil and decreases dramatically as the loose index increases (Figure 3) [40]. For this reason, antlions have evolved a multiscale nonsmooth body surface structure to increase the loose index and reduce the soil excavation resistance.

As the exact formula for calculating the height of a nonsmooth surface bump and the distance between two bumps has rarely been studied in the field of soil mechanics, we borrowed the law of drag reduction from the field of fluids, applied the intrinsic drag reduction mechanism of this law of drag reduction, simplified the complex relationship equation, and applied this principle to the study of this paper in combination with the data obtained on nonsmooth body surfaces of antlion larvae.

It has been shown that nonsmooth surface design could play a role in drag reduction in the field of fluids, and that the same principles of calculating the height of the nonsmooth surface bump and the spacing between the two bumps could be applied to the design of soil-touching components of agricultural machinery [6].

According to the “prominent height” theory in the field of fluid mechanics [41], the groove bump prevents the occurrence of transient crossflow caused by turbulent motion near the wall, and the nonsmooth groove structure leads to a weakening of the turbulent kinetic energy change throughout the boundary layer, thus reducing the viscous drag on the streak surface, as shown in Figure 4, of which the *h*_*ps*_ is the effective protrusion of streamwise direction, and the *h*_*pc*_ is the effective protrusion of the crossflow direction.

According to the gamma and hypergeometric functions [42], the asymptotic equations for the effective protrusion *h*_*p*_ and the riblet height *h* could be expressed as follows. When the cone angle *α* of the raised ribs is kept constant, the following expressions are given, and *S* is the distance between the two bumps.

(1) $$\begin{array}{c} \frac{h_{p}}{s}∼\frac{h}{s}-\tan\left(\alpha /2\right){\left(\frac{h}{s}\right)}^{2}=-\tan\left(\alpha /2\right){\left(\frac{h}{s}-\frac{1}{2\tan\left(\alpha /2\right)}\right)}^{2}+\frac{1}{4\tan\left(\alpha /2\right)}. \end{array}$$

When the *h*/*S* is greater than 1, the approximation formula is to generate an interpolation curve on the asymptote of the blade and the asymptote of the serration, and then the following formula is available, where *ψ* was the Digamma function, which was the logarithmic derivative of the Gamma function.

(2) $$\begin{array}{c} \frac{h_{p}}{s}∼\left(\frac{0.5572}{\pi }\tan\left(a/2\right)+\frac{1}{\pi }\psi \left(1+\frac{\alpha }{\pi }\right)-\frac{1}{\alpha }\tan\left(a/2\right)+1\right)\frac{h}{s}+\frac{\ln2}{\pi }. \end{array}$$

According to Equations (1) and (2), *h*_*p*_/*S* reaches the asymptote when *h*/*S* is between 0.4 and 0.6. When *h*/*S* exceeds 0.6, *h*_*p*_/*S* changes very little.

The article "Bionic Nonsmooth Drag Reduction Mathematical Model Construction and Subsoiling Verification" was published in 2021. Journal: Appl Bionics Biomech.

Based on the “prominent height” theory, the flow state of the fluid is related to *h*, *S*, and the angle of *α*. As *h*/*S* increases, *h*_*p*_/*S* tends to be asymptotic, which indicates that in the design of nonsmooth surfaces, when the size of the moving parts is certain, and the height of the nonsmooth surface increases to a certain degree, the effect of the nonsmooth surface on the fluid flow will gradually become weaker, and the drag reduction effect will stabilize. On the contrary, the nonsmooth surface itself increases the disturbance force on the fluid, which is detrimental to the overall drag reduction effect.

This theory is also compatible with the theoretical model of the Strouhal numbers [43]. The Strouhal numbers *S*_*t*_ are related to the speed of vortex separation. This formula is expressed as follows.

(3) $$\begin{array}{c} S_{t}=\frac{fL}{v}, \end{array}$$

where *f* is the vortex separation frequency, *L* is the characteristic length, and *v* is the fluid velocity. For large *S*_*t*_ (order of magnitude 1), viscosity dominates the fluid; for small *S*_*t*_ (order of magnitude 10^−4^ or less), high velocity dominates the oscillation. This theoretical equation shows the relationship between the frequency of vortex separation and the characteristic length of the moving part and the velocity of the movement. This suggests that in order for a continuous drag reduction effect to be achieved on a nonsmooth surface, the bump spacing design needs to allow for a continuous fluctuating effect on the fluid medium. The drag reduction theory and analysis have been applied for soil-touching components design in this study.

The article "Bionic Nonsmooth Drag Reduction Mathematical Model Construction and Subsoiling Verification" was published in 2021. Journal: Appl Bionics Biomech.

Similar to the theory of drag reduction in fluids with nonsmooth surfaces, the principle of nonsmooth drag reduction in soil is also to allow fluctuations in soil particles, reducing the adhesion of the soil to the touching parts, transforming the soil particles from a single direction of motion to a haphazard motion, and decreasing the adhesion between the soil particles and also between the soil particles and the touching parts, as shown in Figures 5 and 6.

In this research, a friction model between the soil and the soil-touching part was developed in response to the resistance reduction process when the antlions penetrate the soil. Figures 5 and 6 show the soil movement models for smooth and nonsmooth surfaces separately. When the soil-touching part has a smooth surface, it disturbs the soil slightly; the soil remains in its original touching condition; the loose index shows slight variation; there is no drag reduction characteristic (Figure 5).

When the soil-touching part has a nonsmooth surface, the soil fluctuation during the movement is more significant, and the loose index gets bigger. The nearer the area is to the soil-touching part, the more soil fluctuation and the greater loose index is. The layer with a significant change in the loose index is defined as the disturbed layer in this paper (Figure 6). According to the relationship in Figure 3, the internal friction index of the soil in this zone is smaller, and there is less adhesion and frictional resistance during the movement.

In order to express the relationship between the movement of the soil particles and the resistance reduction more clearly, a schematic diagram is made as shown in Figure 7, where the movement of the soil-touching component drives the movement of the soil particles. As the touching part with a nonsmooth surface moves through the soil, the soil particles are disturbed. In the process of returning to its original state, it is subjected to four forces: gravity *G*, support force *F*_*N*_, friction force *F*_*f*_, and adhesion force *F*_*a*_. Due to the complexity of the force changes during the movement of soil particles, the force changes of individual particles are not easy to characterize, and relevant models are less studied. Therefore, in this study, the analogy between the nonsmooth drag reduction of soil-touching components and the drag reduction principle in the fluid field was still made.

When a soil particle is disturbed by a nonsmooth surface, it takes some time to return to its original state. In order to produce a continuous disturbance effect on the soil particle, it needs to be disturbed again before the soil particle returns to its original state. As shown in Figure 7, when the soil particles move with curve 2, it is just enough to achieve a continuous disturbance effect, curve 1 can sufficiently cause soil particles to be disturbed, and curve 3 does not achieve a continuous disturbance effect. In this study, the mechanical model was simplified and combined with the nonsmooth surface structure of the antlion larvae to design the nonsmooth bionic subsoiler shovel tips.

The article "Bionic Nonsmooth Drag Reduction Mathematical Model Construction and Subsoiling Verification" was published in 2021. Journal: Appl Bionics Biomech.

When only the forces in the vertical direction are studied, and assuming that the combined forces on the soil particles after disturbance are of constant value and the acceleration is also of constant value, the following derivative relations are available.

The fluctuating property of the nonsmooth surface increases the loose index of the soil particles. When it comes to a halt, the soil particles return to their original condition from their loose condition, assuming that this recovery time is *t*_*r*_. The amount of this parameter is dependent on the soil class, and the altitude of the nonsmooth surface bulges. In order to acquire a sustainable drag-reducing result, it is necessary to keep the soil particles in a continuous loose condition; the soil should fluctuate twice for a time shorter than the recovery time *t*_*r*_ to obtain the drag-reducing result.

Based on the above analysis, the influencing factors of resistance reduction on nonsmooth surfaces are further quantified. Given that the acceleration for the soil to return from its loose condition to its original condition is *a*, the altitude of the nonsmooth surface bulge is *h*, the movement velocity of the soil-touching part is *v*, the distance between the two bulges is *S*, the time spent by the soil-touching part to travel from one bulge to the other is *T*, and the following equation is obtained.

(4) $$\begin{array}{c} S=v\times T. \end{array}$$

The relationship between bulge altitude and recovery time is as follows:

(5) $$\begin{array}{c} h=\frac{1}{2}\cdot a\cdot t_{r}^{2}. \end{array}$$

In order to ensure the loose condition throughout, recovery time should be greater than the movement period of bulges.

(6) $$\begin{array}{c} t_{r}>T,\text{or }t_{r}=k\cdot T. \end{array}$$

In this equation, the value of *k*, the fluctuation correction index, reaches no less than 1 and is associated with the kind of nonsmooth surface structure.

According to Equations (4)–(6), the acceleration *a* is obtained as follows.

(7) $$\begin{array}{c} a=\frac{2h}{k^{2}T^{2}}=\frac{2hv^{2}}{k^{2}S^{2}}. \end{array}$$

Relationship between the altitude of the bulge *h* and the distance of two bulges *S* is as follows.

(8) $$\begin{array}{c} h=\frac{k^{2}aS^{2}}{2v^{2}}. \end{array}$$

Analysis of the data on the body surface structure of antlions compared with Equation (8) revealed that the altitude of the antlions body bulge was also precisely proportional to the square of the distance between two bulges, but the overall scale factor was slightly different at the three different scales. The reason for this is that the acceleration *a* for the soil to return to its original state differs under variable scale conditions, with the smaller the scale, the greater the acceleration *a*. This is because when the scale decreases, the intermolecular forces are enhanced, accelerating the capability of the soil to return to its original condition. Equation (8) can be used for the design of subsoiler shovel tip, and the meaning and basis for determining each parameter are summarized in Table 1.

The article "Bionic Nonsmooth Drag Reduction Mathematical Model Construction and Subsoiling Verification" was published in 2021. Journal: Appl Bionics Biomech.

Natural organisms have evolved over billions of years and have become highly adaptable to their environment. And the nonsmooth body structure of the antlion larvae has been shown to correlate with their rapid burrowing in the soil [26]. This suggests that the antlion larvae have evolved a body structure which is well adapted to the soil environment, and its nonsmooth body surface structure contributes to a continuous fluctuation of the soil. Assuming that the nonsmooth body surface structure of the antlion larvae is just sufficient to cause a continuous disturbance of the soil, the acceleration at which the soil returns to its original state at different nonsmooth surface scales of the antlion larvae is back-calculated according to Equation (7), as shown in Table 2.

### 2.3. Subsoiler Shovel Tip Design

Based on the nonsmooth drag reduction mathematical model, type B and type E subsoiler shovel tips were designed, as shown in Figure 8.

Types A, B, and C are flat shovel tips with a width of 150 mm, a tip angle of 60°, and a thickness of 10 mm. Type A has a smooth shovel surface; type C is the control group and is a subsoiler shovel tip imitating pangolin scales. Types D, E, and F are upconvex curved shovel tips, and the other parameters correspond to types A, B, and C one by one (Table 3).

The equation for the rib curves on the subsoiler shovel tips B and E is as follows.

(9) $$\begin{array}{c} y=-0.0051x^{3}-0.0474x^{2}+1.0089x+0.2105. \end{array}$$

Equation (9) was obtained by a three-dimensional scan of the antlion larvae's overall structure. The antlion larvae back's maximum profile curve of the longitudinal profile was extracted, fitted, and then reasonably enlarged in size, with a fitted correlation coefficient of *R*^2^ = 0.9541 and a range of values for *x* in Equation (9), *x* ∈ [−0.5, 10.5]. The graph enclosed by this curve and the *x*-axis straight line were used as the cross-section of the shovel tips body bionic structure and were welded to the shovel tip substrate. The designed curve covered the body of the shovel tip. The spacing between the ribs on tips B and E was 17 mm, the radius of the hemispherical projection of the tips was 2 mm, the transverse spacing was 6 mm, and the longitudinal spacing was 7 mm. The radius of curvature of tips D, E, and F was 300 mm, the scales on tips C and F were closely spaced, the individual scales were wedge-shaped, and the maximum thickness was 2 mm.

The article "Bionic Nonsmooth Drag Reduction Mathematical Model Construction and Subsoiling Verification" was published in 2021. Journal: Appl Bionics Biomech.

## 3. Field Experiment Validation

### 3.1. Soil Testing

The soil environment is an important indicator influencing the subsoiling testing and needs to be tested before the experiments [44]. The field experiments were carried out at the Tongqing Village, Taojiatun Town, Gongzhuling City, Jilin Province, China (125.0°E, 43.6°N). The soil moisture contents were obtained from a soil moisture sensor (Spectrum TDR 300, America). Ten random sampling points were measured at each soil depth condition, and the variation of water content with depth in the test field is shown in Figure 9. The average water content ranged from 24.7% to 42.0% at depths from 0 cm to 50 cm.

A soil particle size distribution at different depths was tested by a laser particle size analyzer (XF3000); samples were taken at five sampling points, and the test results were averaged to obtain the soil particle size distribution as shown in Table 4. According to the international standard soil type classification [10], the soil in the test area belongs to loamy soil in the depth range of 0-40 cm and powdered sandy loam in the depth range of 40-50 cm.

### 3.2. Field Experiments

The test field was selected from a postharvest maize field (Figure 10), and three operating speeds (3 km/h, 5 km/h, 7 km/h) were chosen according to the tillage range. The operating speed was able to be displayed on the tractor panel and could be controlled by the accelerator pedal and gears. The depth of subsoiling was divided into three types, which were 30 cm (typical depth), 20 cm, and 40 cm. The tractor was operated for 100 m at each desired speed, and each test was repeated three times. The first ten meters were used to adjust the tractor's working depth and speed for a steady distance of eighty meters, and the last ten meters were used to gradually reduce the speed and stop.

### 3.3. Measurements

#### 3.3.1. Subsoiling Resistance

Subsoiling resistance was tested with a field resistance dynamometer (Harbin, China), which consisted of upper suspension sensors, lower suspension sensors, a data acquisition tool, inclination sensors, and a receiver. The upper and lower suspension sensors were hooked up to three attachment points on the tractor. Each sensor had a measuring range of 15 kN and a sensitivity of 0.045 kN. The sensor input voltage was 24 V DC, and the output current was 20 mA. The resistance values measured by the sensors were sent through wireless to a computer. The subsoiler was mounted on the frame, and the subsoiler shovel tips were all mounted on the same universal shovel handle, so that the subsoiling resistance could be transmitted directly to the three force sensors. The subsoiler shovel tips were mounted on the shovel handle of the Chinese national standard type by two screws for easy removal and were fixed to the frame by screws.

The article "Bionic Nonsmooth Drag Reduction Mathematical Model Construction and Subsoiling Verification" was published in 2021. Journal: Appl Bionics Biomech.

#### 3.3.2. Soil Penetration Resistance

Soil penetration resistance was measured with a penetration resistance measurement instrument (Spectrum TDR 300, America), which tested the firmness values before subsoiling and after subsoiling at the bottom of the trench and 30 cm from the bottom of the trench, respectively. Measurements were taken at a depth of 45 cm, with samples taken every 25 mm, and five replicate tests were carried out for each test.

## 4. Results and Discussion

In this section, the resistance values of six subsoiler shovel tips at three different speeds and depths were compared to verify the effect of the shovel tips (tips B and E) designed with a mathematical model to reduce drag and to explain the principle of drag reduction. Changes in soil firmness before and after subsoiling were compared to assess the effect of subsoiling on the soil environment.

### 4.1. Analysis of the Subsoiling Resistance

Figures 11–13 show the variation of traction force with operating distance for the six subsoiler shovel tips at a subsoiling depth of 30 cm, at three speeds of 3 km/h, 5 km/h, and 7 km/h. The stabilized traction force values of the six subsoilers at three speed conditions were chosen and averaged under three replicate tests (Figure 14). The relationships between the different parameters of the field experiments were analyzed below. In this study, each experiment was repeated five times, and only the median resistance for the five replicated experiments was shown in Figures 11–13.

#### 4.1.1. Effect of Subsoiler Shovel Tip Type on Subsoiling Resistance

The type of subsoiler shovel tip had a significant effect on the subsoiling resistance. Combining the three speeds and comparing subsoiler shovel tip D, tip E, and tip F, tip E had the lowest resistance, tip F the second lowest, and tip D the highest. Compared to tip D, tip E could reduce resistance by an average of 24.6%, and tip F could reduce resistance by 16.9%. Compared with tip A, tip B, and tip C, tip B could reduce resistance by 19.34% and tip C by 16.14% on average compared with tip A. In this experiment, the subsoiler shovel tip E designed according to the mathematical model showed a good drag reduction effect, because the contact between the soil and the shovel tip surface was changed through surface reshaping. The nonsmooth shovel surface caused soil particle disturbance during movement, increasing the soil loose index, especially in the area closer to the soil-touching part, showing that the greater the loose index was, the less soil adhesion and drag became. Comparing tip E and tip F, tip E had a more significant drag reduction effect, indicating that the modeled nonsmooth surface had a greater drag reduction capacity.

The article "Bionic Nonsmooth Drag Reduction Mathematical Model Construction and Subsoiling Verification" was published in 2021. Journal: Appl Bionics Biomech.

Comparing tip D, tip E, and tip F with tip A, tip B, and tip C, the upper convex surface had a lower resistance, with a maximum of 9.1% reduction in subsoiling resistance. The upper convex curved subsoiler shovel tip could deflect the soil on both sides during the subsoiling process, making it less likely to form soil nuclei and reduce resistance. The results of the six types of subsoiler shovel tips at three speeds and a depth of 30 cm showed that the curved shovel tip E designed according to the model had the most significant drag reduction effect, with a drag reduction rate of 24.6%.

#### 4.1.2. Effect of Depth on Subsoiling Resistance

The depth of subsoiling had an enormous impact on the resistance. The resistance of subsoiling is mainly generated by several forces on soil lifting, compression, shear, and friction. When the depth increases, the pressure of the subsoiler on the soil increases; all these forces will increase and therefore, the resistance increases. Figures 15 and 16 show the resistance of the six subsoiler shovel tips at 20 cm and 40 cm depths, respectively. Comparing the resistance data for a subsoiling depth of 30 cm, the resistance values decreased by an average of 27.37% for the 20 cm depth condition and increased by an average of 23.06% for the 40 cm depth.

Comparing the resistance performance of the six subsoiler shovel tips at three speeds, the nonsmooth surface also showed a good reduction ability in resistance. At a depth of 20 cm, tip E reduced drag by 30.49%, and tip F reduced drag by 17.10% compared to tip D; at a depth of 40 cm, tip E reduced drag by 33.72%, and tip F reduced drag by 17.40%. Further validating the effect of nonsmooth surfaces, the curved tip E obtained from the model also showed more significant drag reduction, with 30.49% at 20 cm depth and 33.72% at 40 cm depth.

#### 4.1.3. Effect of Operating Speed on Subsoiling Resistance

In this study, the subsoiling resistance increased slightly but not significantly with the increase in operating speed. The reason for this might be that under the soil conditions, the flow state of the soil on the subsoiler shovel tip face was better, and the squeezing effect of the subsoiler shovel tips in the soil on both sides was not significantly enhanced when the speed was increased, resulting in an insignificant increase in subsoiling resistance.

The article "Bionic Nonsmooth Drag Reduction Mathematical Model Construction and Subsoiling Verification" was published in 2021. Journal: Appl Bionics Biomech.

Comparing the resistance values of the tip E at different speeds, it could be seen that the subsoiling resistance of the tip E tended to decrease as the speed increased, which was because the nonsmooth surface structure on the tip E could cause more effective soil disturbance and achieve better drag reduction effect as the speed increased, further verifying the correctness of the mathematical model established in this study.

### 4.2. Changes in Soil Firmness before and after Subsoiling

The change in soil firmness is one of the most important indicators of subsoiling effectiveness. In this study, in order to verify the effect of subsoiling with the subsoiler shovel tip E, the change in soil firmness before and after subsoiling was tested at a depth of 30 cm and a speed of 3 km/h. Before subsoiling, the soil firmness tended to increase and then decrease with depth, with the maximum value occurring between 20 and 30 cm (Figure 17), which was the area at the plow pan. The soil firmness values dropped sharply after the subsoiling, with the most pronounced drop in soil firmness at the bottom of the subsoiling furrow. In this experiment, the spacing between the two subsoiling operations was 60 cm; thus, the area showing minimum disturbance was 30 cm from the subsoiling furrow. In this area, the soil firmness dropped sharply, indicating that the subsoiling operation had achieved good results. Compared with the soil firmness at 25 cm depth, the soil firmness decreased by 63.5% at a depth of 30 cm from the subsoiling furrow after subsoiling, indicating that the nonsmooth curved subsoiler shovel tip designed according to the mathematical model in this study not only had the effect of reducing resistance but also could achieve the effect of overall subsoiling.

## 5. Conclusions

In this study, the mechanism of nonsmooth surface drag reduction was analyzed, the relationship between the altitude of the nonsmooth drag-reducing surface bulge, the distance between the bulges, and the movement speed was deduced, a nonsmooth drag-reducing surface design mathematical model was established, and the correctness of the model was verified through subsoiling experiments in the field.

The drag reduction effect of the nonsmooth subsoiler shovel tips was generally lower than that of the flat subsoiler shovel tips, and the drag reduction effect of the subsoiler shovel tips designed according to the model was better. At different depths, the drag reduction rate of the curved subsoiler designed according to the model reached 24.6% to 33.7%; with the increase of subsoiling depth, subsoiling resistance ascended obviously; operation speed contributed to improving the drag reduction effect of nonsmooth surface and had no obvious effect on subsoiling resistance. The modeled curved surface subsoiler shovel tip had an overall subsoiling effect on the soil.

The article "Bionic Nonsmooth Drag Reduction Mathematical Model Construction and Subsoiling Verification" was published in 2021. Journal: Appl Bionics Biomech.

In this research, the subsoiler shovel tip obtained by the model of nonsmooth drag-reducing surface design showed a good drag-reducing effect in the filed subsoiling experiments, which was of great significance for the design of soil touching parts' nonsmooth drag-reducing surface.

## Figures and Tables

**Figure 1:** Antlions surface structure of the whole body. (a) The whole body. (b) Tip of jaw. (c) Jaw. (d) Magnified view of margin. (e) Marginal structure. (f) Head. (g) Back. (h) Tail setae. (i) Magnified view of tail. (j) Tail.

**Figure 2:** Correspondence between positive stress, soil shear force, and angle of internal friction [40].

**Figure 3:** Correspondence between internal friction index and loose index [40].

**Figure 4:** The “prominent height” theory.

**Figure 5:** Smooth surface soil friction model.

**Figure 6:** Model of soil movement on nonsmooth surfaces.

**Figure 7:** Schematic diagram of the individual soil particle movement.

**Figure 8:** Six types of subsoiler shovel tips.

**Figure 9:** Variation of water content with depth.

**Figure 10:** Subsoiling field experiments.

**Figure 11:** Variation of subsoiling resistance with distance for six subsoilers at 3 km/h speed and 30 cm depth.

**Figure 12:** Variation of subsoiling resistance with distance for six subsoilers at 5 km/h speed and 30 cm depth.

**Figure 13:** Variation of subsoiling resistance with distance for six subsoilers at 7 km/h speed and 30 cm depth.

**Figure 14:** Mean values of subsoiling resistance for six types of subsoilers at three speeds and 30 cm depth.

**Figure 15:** Mean values of subsoiling resistance for six types of subsoilers at three speeds and 20 cm depth.

**Figure 16:** Mean values of subsoiling resistance for six types of subsoilers at three speeds and 40 cm depth.

**Figure 17:** Variation in soil firmness with depth before and after subsoiling.

**Table 1:** Meaning and basis for determining the parameters.

Parameters	Meaning	Basis of determination
*h*	Altitude of bulge	Minimum value causing effective soil fluctuations
*S*	Bulge spacing	Determined by the altitude of the bulge *h*
*v*	Movement speed	Movement speed of the soil-touching part
*a*	Acceleration	Decreasing with increasing scale of soil-touching part
*t*_*r*_	Recovery time	Determined by acceleration *a*
*T*	Cycle time	Time to move one pitch of bulge
*k*	Correction index	Associated with nonsmooth surface morphological features

The article "Bionic Nonsmooth Drag Reduction Mathematical Model Construction and Subsoiling Verification" was published in 2021. Journal: Appl Bionics Biomech.

**Table 2:** The acceleration of soil restoration to its original state at different scales.

Acceleration (m/s^2^)	Back and abdomen submillimeter protrusions/edge bristles	Back/abdomen/head/tail bristles	Back/abdomen submicron structure
$a=\frac{2h}{T^{2}}=\frac{2hv^{2}}{S^{2}}$	0.34	3.24	4.11

**Table 3:** Subsoiler shovel tip design.

Flat surface			Curved surface		
A	B	C	D	E	F
Smooth tips	Mathematical model tips	Pangolin bionic tips	Smooth tips	Mathematical model tips	Pangolin bionic tips

**Table 4:** Soil particle size distribution at different depths.

Sampling depth (cm)	Percentage mass of soil particle size distribution at each level (%)		
	Viscous particles (less than 2 *μ*m)	Powdered sand particles (2 *μ*m-20 *μ*m)	Sand particles (20 *μ*m-2 mm)
0-10	7.74	38.69	53.57
10-20	9.21	36.83	53.96
20-30	9.39	35.74	54.87
30-40	10.85	41.17	47.98
40-50	12.02	45.18	42.80

## Data Availability

The data used to support the findings of this study are available from the corresponding author upon request.
